The article "A Machine Learning Model to Predict Citation Counts of Scientific Papers in Otology Field" was published in 2022. Journal: Biomed Res Int.

# A Machine Learning Model to Predict Citation Counts of Scientific Papers in Otology Field

**DOI:** 10.1155/2022/2239152

**Published:** 2022-07-20

**Authors:** Yousef A. Alohali, Mahmoud S. Fayed, Tamer Mesallam, Yassin Abdelsamad, Fida Almuhawas, Abdulrahman Hagr

**Affiliations:** ^1^College of Computer and Information Sciences, King Saud University, Riyadh, Saudi Arabia; ^2^Research Chair of Voice, Swallowing and Communication Disorders, Department of Otorhinolaryngology-Head and Neck Surgery, King Saud University, Riyadh, Saudi Arabia; ^3^Research Department, MED-EL GmbH, Riyadh, Saudi Arabia; ^4^King Abdullah Ear Specialist Center (KAESC), College of Medicine, King Saud University, Riyadh, Saudi Arabia

## Abstract

One of the most widely used measures of scientific impact is the number of citations. However, due to its heavy-tailed distribution, citations are fundamentally difficult to predict but can be improved. This study was aimed at investigating the factors and parts influencing the citation number of a scientific paper in the otology field. Therefore, this work proposes a new solution that utilizes machine learning and natural language processing to process English text and provides a paper citation as the predicted results. Different algorithms are implemented in this solution, such as linear regression, boosted decision tree, decision forest, and neural networks. The application of neural network regression revealed that papers' abstracts have more influence on the citation numbers of otological articles. This new solution has been developed in visual programming using Microsoft Azure machine learning at the back end and Programming Without Coding Technology at the front end. We recommend using machine learning models to improve the abstracts of research articles to get more citations.

## 1. Introduction

In the research world where researchers publish the results of their work through research papers, one can consider the paper citations as one of the common indicators of the paper's quality, importance, and relevance. This is in contrast to the software world where its success is measured by the number of downloads or to the social media world, like Facebook posts and YouTube videos, where the number of views/interactions is the major Key Performance Indicator (KPI) beside the scientific content of research articles; other factors influence the paper citations like social effects, author's name, and the journal rank [1, 2].

Most academic papers are scarcely cited while a few others are highly cited. Some factors such as the paper's quality, journal impact, number of authors, visibility, and international cooperation are stronger predictors than others such as authors' gender, age, and race and characteristics of results and discussion [3]. Moreover, as citations demonstrate a heavy-tailed distribution, with most publications receiving few citations, these simple measures are exceedingly difficult to estimate using traditional regression analysis [4, 5].

Citation prediction of scholarly papers is of great significance in guiding funding allocations, recruitment decisions, and rewards. Models use multifeatures predictive through author-based, journal-based, and citation [6]. Funding agencies and researchers with limited time and resources increasingly seek metrics and models to quantify the potential impact of a collaboration or a proposal [7–9].

The remainder of this paper is organized as follows.  Section 2 describes related works.  Section 3 illustrates the dataset.  Section 4 demonstrates using machine learning to implement the different models.  Section 5 presents experimental results and analysis, while Section 6 demonstrates the Ring programming language and the Programming Without Coding Technology tool to build the citation prediction application and a user interface. Finally, we present the discussion, future work, and the conclusion in Section 7.

## 2. Related Work

In [10, 11], Newman conducted a study based on finding the relationship between the publication date, topic, and an early number of citations. He identified several papers that could have a high impact in the future. In a dataset of 2000 papers, he expected that 50 papers will do the best. After five years, on average these papers received 23 times as many citations as the initial count and 15 times as many as the average paper in a randomly drawn control group that started with the same number of citations.

In [12], Dong et al. used statistical methods to know if the paper will increase the *h*-index. They studied the correlation between the citations and many factors related to the paper's author, content, venue, social, and references.

In [13], the authors used a neural network to predict the citations based on features like paper ID, title, author score, number of published papers by the author, average download rates, and average number of citations for the author.

In [14], the authors presented a study on biomedical research papers, they built a model using support vector machines (SVMs) using features like title, abstract, number of articles (for the first author), number of citations (for the first author), number of articles (for the last author), number of citations (for the last author), publication type, number of authors, number of institutions, and journal impact factor.

In [15], the authors developed a machine learning model and a web-based *h*-index predictor using the author *h*-index, total publications, and the absolute year of the first publication by the author. Also, the application support prediction uses paper information like title, authors, year, and abstract. The dataset contains 1,712,433 authors with 2,092,356 papers from computer science venues held until 2012. They used logistic regression (LRC), support vector machine (SVM), naive Bayes (NB), radial basis function network (RBF), bagged decision trees (BAG), and random forest (RF).

In [16], a dataset containing 1086 papers from the Bioinformatics journal was used. The authors used Bayesian networks (naive Bayes and K2), logistic regression, decision trees, and the *K*-nearest neighbor (K-NN) algorithm to predict the citations. The accuracy of naive Bayes and logistic regression supervised classification methods was 89.4% and 91.5%, respectively.

In [17], the authors used a dataset containing 8 million bibliographic entries spanning over 3 million unique authors. They used Shannon entropy and Jensen-Shannon divergence to model the effects of each author's influence and the words in the title of the paper. They used naive Bayes, logistic regression, support vector machine (SVM), random forest, and boosted trees and achieved an accuracy of 88%.

In [18], the authors used multivariate analyses in three journals in the field of social-personality psychology. They discovered that the author's gender and nationality, collaboration, and university prestige do not predict the impact. But the first author's eminence, journal prestige, and article length predict the impact.

Research about the impact of scientific articles mainly focuses on two interrelated questions: how to assess the past impact of an article and how to accurately predict its future impact. This includes using techniques like quantile regression, multivariate analysis, multivariate analysis random forest classifier long term, correlation analysis, and linear regression analysis [19]. Some of the open challenges could include sleeping beauty, multidimensional prediction, and rising star prediction [20, 21].

In [22], the authors used a dataset of 38 million papers and 19 million authors. They focus on publications dated from 2000 to 2005 in seven key domains (12.7 million papers and 3 million authors). The domains are CS, biology, chemistry, medicine, engineering, mathematics, and physics. They used features like authors, institutions, venues, reference network (citations), and content similarity. They used a support vector regression machine (SVR) model, and the achieved accuracy varies between 17% and 39% based on the domain. The accuracy of the prediction is calculated using the *R*-squared of the predictions with actual citations. The *R*-squared (coefficient of determination) evaluates the scatter of the data points around the fitted regression line.

In [23], the authors discovered the association between two variables and the paper citations. These variables are the sum of repetition of keywords in abstract divided by abstract length and the frequency of paper's keyword per journal. These results are based on using a dataset of 5875 papers from 12 journals in the education.

In [24], the authors did a study that proves that journals that publish papers with shorter titles receive more citations per paper. In [25], the authors did another study that proves that articles with short titles describing the results are cited more often.

In [26], the authors did a study using a dataset of 6122 papers related to environmental modeling. They used features like citation count, year, page count, author count, author name, journal, abstract length, title length, and special issue. They discovered that the number of citations could be predicted with no knowledge about the paper quality.

Scientific breakthroughs are rare events. In [27], the authors developed methods that combine curve fitting and thresholding strategies for the early detection of candidate breakthrough papers.

In [28], the authors discovered that the BP neural network significantly outperformed the other six baselines (XGBoost, RF, LR, SVR, KNN, and RNN).

In [29, 30], the authors showed that a wide range of descriptors is necessary as an input to the machine learning algorithms, such as decision forest and neural networks, for improved accuracy. These studies [29, 30] used input descriptors to describe the chemical molecular in 3D space (i.e., molecular descriptors). In this study, since the input is a text written in the English language, we used natural language processing as a stage that processes the text and produces such descriptors.

From the previous studies, we notice that the paper citation prediction results are different based on the following:

(i) The dataset used (domain and size): very large datasets are more general but lead to low prediction accuracy compared to small and specialized datasets.
(ii) The change in the features used in the prediction will lead to different results, and feature selection plays an important role.
(iii) Many machine learning models could be used, and the performance of each model is different based on the dataset and used features.
(iv) The user who will benefit from the citation prediction applications could be the following:
  - Paper author: who wants to improve his/her paper
  - Journal editor: who wants to accept the best papers
  - Researcher: who wants to select which papers to read.

So developing a custom solution for each domain could provide the best benefit for the interested researchers. This process should include using a custom dataset, doing the right feature selection, and testing different machine learning models to use the best one that provides the highest level of accuracy.

## 3. The Dataset

Our dataset contains 500 research papers (500 rows)—we have information about each paper like the title, authors, abstract, and total citations.

For the total citation (TC) column, the minimum value is 57 citations, while the maximum value is 579 citations. So we have a range of 579‐57 + 1 citations, i.e., 523 citations.

The dataset is available as a PDF file, and we saved the file as a text file (using the “Save As” feature from the Acrobat PDF reader); then, we converted the TXT file to a CSV file using a program written in the Ring programming language [31]. This Ring program is generated using the Programming Without Coding Technology (PWCT) software which is considered a general-purpose visual programming language [32–34]. PWCT is a popular visual programming language that is used in many applications and systems including the development of the Supernova language and the critical node application for the LASCNN algorithm [35, 36].

## 4. Algorithms and Machine Learning Models

### 4.1. Algorithms

This study uses the next algorithms for regression. We picked some of the popular machine learning algorithms in the literature [37–39].

- Linear regression
- Boosted decision tree regression
- Decision forest regression
- Neural network regression

The next tools are used for development.

- Microsoft Azure machine learning: we selected this tool because it is a visual tool that supports many machine learning models and reduces the development time [40–42].
- The Ring programming language: we selected this language because it is a simple and dynamic programming language like Python but comes with integrated GUI tools like Visual Basic
- Programming Without Coding Technology (PWCT): we selected this tool because it is a visual programming language that reduces development time

Steps:

- Prepare and analyze the dataset
- Preprocess the text
- Split the data (training data and test data)
- Extract *n*-gram features
- Select columns
- Select the algorithm
- Train the models
- Score and evaluate (calculate the root mean squared error)
- Compare the results between the different algorithms

### 4.2. Natural Language Processing

Preprocess text: in this stage, the text is processed before usage by our machine learning model.

- Remove stop words
- Preform lemmatization
- Detect sentences
- Normalize case to lowercase
- Remove numbers
- Remove special characters
- Remove duplicate characters
- Remove email addresses
- Remove URLs
- Expand verb contraction
- Split tokens on special characters

Split data: 70% of our data is used for training while 30% is used for testing.

#### 4.2.1. Extract *n*-Gram Features

There are many weighting functions like binary weight, TF weight, IDF weight, TF-IDF weight, and graph weight. In this stage, we used the TF-IDF weighting function. The minimum word length is three (3) while the maximum word length is 25. The minimum *n*-gram document absolute frequency is five (5). The maximum *n*-gram document frequency ratio is 80%. There are many feature scoring methods like Pearson correlation, mutual information, Kendall correlation, Spearman correlation, chi-squared, fisher score, and count based. The feature scoring method used in our experiments is chi-squared.

## 5. Experimental Results and Analysis

### 5.1. Prediction Using the Title

Concerning the maximum *n*-grams in the model parameters, we allowed 2000 *n*-grams. In practice, the model uses 165 columns including 164 *n*-grams. The other column is the total citations.  Table 1 provides some of the *n*-grams used by the model and their weight.

Some of the *n*-gram have positive weight, while other *n*-gram have negative weight as demonstrated in Table 2.

In Figure 1, the word art visualizes the *n*-gram features. From this figure, we notice that some words come with big weight (more importance) like ganglion, speak the language, and chronic. The figure uses the font size, location, and colors to demonstrate the importance of the word.

Table 3 provides the results when predicting the total citations using the title.

In this experiment, the decision forest regression provides the minimum root mean squared error (69.45); then, we have the boosted decision tree regression providing the root mean squared error (70.15) while the linear regression provides 80.43 as the root mean squared error, and finally, the neural network provides 87.51 as the root mean squared error. So, in this case, the best algorithm is the decision forest regression.

The dataset contains 500 papers; out of these papers, we have 350 papers used for training and 150 papers used for testing (using the decision forest regression). The citation range is 523 citations.

Table 4 demonstrates the error percentage while predicting the citations for 150 papers during the testing stage.

Table 4 is a good indicator of the model's accuracy. If we considered that the error in citation prediction should be less than 40 citations (7.6% of the citation range), then we have 65.33% of papers passing this condition. Considering that the error should be less than or equal to 100 citations (19.12% of citation range), then 87.33% of the papers in the testing stage pass this condition.

Figure 2 demonstrates the root mean squared error for different models using the title *n*-grams.

### 5.2. Prediction Using the Abstract

Concerning the maximum *n*-grams in the model parameters, we allowed 2000 *n*-grams. In practice, the model uses 1715 columns including 1714 *n*-grams. The other column is the total citations.

Table 5 provides some of the *n*-grams used by the model and their weight.

Table 6 demonstrates that some of the *n*-grams have positive weight, while other *n*-grams have negative weight.

In Figure 3, the word art visualizes the *n*-gram features; from this figure, we notice that some words like specimen and chronic have higher weight and are more important.

Table 7 presents the next results when predicting the total citations using the abstract.

In this experiment, the neural network provides the minimum root mean squared error (62.76); then, we have the decision forest regression providing the root mean squared error (63.53) while the boosted decision tree regression provides 66 as the root mean squared error, and finally, the linear regression provides 68.56 as the root mean squared error. So, in this case, the best algorithm is the neural network.

The dataset contains 500 papers; from these papers, we have 18 papers that come without abstracts. We have 337 papers used for training and 145 papers used for testing (using the neural network regression). The citation range is 523 citations.

Table 8 demonstrates the error percentage while predicting the citations for 145 papers during the testing stage.

Table 8 is a good indicator of the model's accuracy. If we considered that the error in citation prediction should be less than 40 citations (7.6% of the citation range), then we have 64.13% of papers passing this condition. Considering that the error should be less than or equal to 100 citations (19.12% of citation range), then 93.1% of the papers in the testing stage pass this condition.

Figure 4 demonstrates the root mean squared error for different models using the abstract *n*-grams.

### 5.3. Prediction Using the Authors

For the maximum *n*-grams in the model parameters, we allowed 2000 *n*-grams. In practice, the model uses 95 columns including 94 *n*-grams. The other column is the total citations.

Some of the *n*-grams have positive weight, while other *n*-gram has negative weight.

Table 9 provides the results when predicting the total citations using the authors.

In this experiment, the boosted decision tree regression provides the minimum root mean squared error (65.79); then, we have the decision forest regression providing the root mean squared error (67.36) while the linear regression provides 69.58 as the root mean squared error, and finally, the neural network provides 70.19 as the root mean squared error. So, in this case, the best algorithm is the boosted decision tree regression.

The dataset contains 500 papers; one paper comes without the authors. We have 349 papers used for training and 150 papers used for testing (using the boosted decision tree regression). The citation range is 523 citations.  Table 10 demonstrates the error percentage while predicting the citations for 150 papers during the testing stage.

Table 10 is a good indicator of the model's accuracy. If we considered that the error in citation prediction should be less than 40 citations (7.6% of the citations range), then we have 60% of papers passing this condition. Considering that the error should be less than or equal to 100 citations (19.12% of citations range), then 90.66% of the papers in the testing stage pass this condition.

Figure 5 demonstrates the root mean squared error for different models using the author *n*-grams.

### 5.4. Web Services

We published a web service for each trained model (boosted decision tree, decision forest, and neural networks).

## 6. Citation Prediction Application

We developed an application that can accept the title, authors, and abstract to predict the total citations (demonstrated in Figure 6). The application is developed using the Ring programming language where the source code is generated using the Programming Without Coding Technology (PWCT) software. The main window in our application provides a data entry form that we can use to enter the paper details. We need at least to determine the title, author, or abstract. Then, we click the “Predict” button to get the prediction results. Using the “Select” button, we get another window that contains our dataset rows, where we can quickly select any of these rows and use them for testing our application.

Figure 7 presents the dataset rows; each row in our dataset contains the three features (title, authors, and abstract) and one label (total citations). The title, authors, and abstract are textual data while the total citations are numeric data.

We can select a row and then click on the “Select” button to insert the row data in our main window as demonstrated in Figure 8.

## 7. Discussion, Future Work, and Conclusion

### 7.1. Discussion and Future Work

The results of these research and case studies demonstrate that we can use different machine learning algorithms to build models that predict the paper citations using different features. We detected the best algorithm for the different features like the title, authors, and abstract. The difference in RMSE between the algorithms when using the same feature is not so big, but the difference in RMSE when using the different features could be notable. The best result could be achieved when using the paper abstract in the prediction.

Table 11 provides each feature, the best algorithm, and the root mean squared error achieved in our experiments while predicting the total citations.

Prediction using the abstract and the neural network provides the minimum root mean squared error (62.76) as demonstrated in Figure 9.

Table 12 provides the used feature and the number of *n*-grams. The graph in Figure 10 presents these results; we notice that when using the abstract feature in the prediction, we have a huge number of *n*-grams.

The predicted paper citation is just an indicator that can be used by the reviewers on the journal side to pick the paper that could be more attractive to the readers. Also, it can be used by the authors of the research to improve the paper's impact by rewriting the paper title and abstract until getting the higher possible prediction of the paper citations.

In the future, we will extend our experiments; for example, we will try more neural networks with different scripts that set the layer count, nodes in each layer, and different activation functions. Also, we plan to try different weight functions in the text processing stage. We plan also to use ensemble learning and use many different models together in the prediction process to get higher accuracy. An improvement that we plan to do too is developing a tool that provides a simple GUI to analyze the prediction output and provide suggestions about which words to keep and which words to change. We plan also to replace our desktop front end application with web-based solution to quickly deliver new updates and a mobile application to have more accessible software.

### 7.2. Conclusion

The use of models that can predict which citations an article will receive after publication can be a useful tool in the publisher's evaluation process. Also, it can help the research authors to improve the paper content to get more citations.

In this paper, we presented a machine learning model to predict the total number of citations of the research papers using different algorithms like boosted decision tree, decision forest, and neural networks. We did many experiments to evaluate the performance of each model and determine which one provides the best results. Our results demonstrate that using neural networks and the paper abstract provides the minimum root mean squared error compared to using other algorithms like the boosted decision tree or the decision forest. We developed the model using the Microsoft Azure machine learning tool and also developed an application using the Programming Without Coding Technology that displays the dataset and predicts the paper citations using different algorithms.

The quality of the research papers could be improved through the adoption of machine learning models by more researchers Also, these models could become more suitable in the future when different machine learning methods and specific datasets could be used for each scientific domain.

## Figures and Tables

**Figure 1:** Title *n*-gram word art.

**Figure 2:** RMSE for different models that use the title *n*-grams.

**Figure 3:** Abstract *n*-gram word art.

**Figure 4:** RMSE for different models that use the abstract *n*-grams.

**Figure 5:** RMSE for different models that use the author *n*-grams.

**Figure 6:** Citation prediction application: main window.

**Figure 7:** Citation prediction application: dataset window.

**Figure 8:** Inserting data from the dataset window to the main window.

**Figure 9:** Graph demonstrates the RMSE achieved by each algorithm.

**Figure 10:** Graph demonstrated the number of *n*-grams for each feature.

**Table 1:** Some of the title *n*-grams with positive weight.

Feature	Weight
Preprocessed TI.[ganglion]	915.36
Preprocessed TI.[speak_language]	188.11
Preprocessed TI.[chronic]	180.89
Preprocessed TI.[ear]	175.04
Preprocessed TI.[implantation]	141.14
Preprocessed TI.[acoustic_stimulation]	138.86
Preprocessed TI.[implication_cochlear]	110.82
Preprocessed TI.[perception_cochlear]	94.83
Preprocessed TI.[adult_use]	86.15
Preprocessed TI.[affect]	78.60
Preprocessed TI.[auditory_nerve]	73.73
Preprocessed TI.[development]	72.84
Preprocessed TI.[language_development]	70.51
Preprocessed TI.[use_cochlear]	66.22
Preprocessed TI.[deafness]	55.75
Preprocessed TI.[skill]	53.03
Preprocessed TI.[electrical]	47.46
Preprocessed TI.[depth]	45.88
Preprocessed TI.[speak]	42.75

**Table 2:** Some of the title *n*-grams with negative weights.

Feature	Weight
Preprocessed TI.[electrode_insertion]	-90.47
Preprocessed TI.[assessment]	-90.87
Preprocessed TI.[profound]	-92.07
Preprocessed TI.[stimulation_auditory]	-93.67
Preprocessed TI.[study]	-94.31
Preprocessed TI.[ganglion_neuron]	-96.39
Preprocessed TI.[implant_patient]	-99.88
Preprocessed TI.[nerve]	-103.80
Preprocessed TI.[congenital]	-106.46
Preprocessed TI.[early_cochlear]	-161.79
Preprocessed TI.[cochlear_implantation]	-164.26
Preprocessed TI.[child_use]	-172.33
Preprocessed TI.[implant_user]	-172.34
Preprocessed TI.[spiral]	-453.88
Preprocessed TI.[spiral_ganglion]	-453.88

**Table 3:** Using different models to predict the total citations using the paper title.

Algorithm	Mean absolute error	Root mean squared error	Relative absolute error	Relative squared error	Coefficient of determination
Linear regression	58.73	80.43	1.21	1.41	-0.41
Boosted decision tree regression	48.67	70.15	1.00	1.07	-0.07
Decision forest regression	46.12	69.45	0.95	1.05	-0.05
Neural network	60.23	87.51	1.24	1.67	-0.67

**Table 4:** Error in citation count.

Error	Percentage of citation range (523 citations)	Papers count	Percentage of testing papers (150 papers)
≤10 citations	1.9%	29 papers	19.33%
≤40 citations	7.6%	98 papers	65.33%
≤80 citations	15.29%	125 papers	83.33%
≤100 citations	19.12%	131 papers	87.33%

**Table 5:** Some of the abstract *n*-grams with positive weights.

Feature	Weight
Preprocessed AB.[specimen]	215.01
Preprocessed AB.[chronic]	201.60
Preprocessed AB.[expression]	188.20
Preprocessed AB.[individual]	180.01
Preprocessed AB.[largely]	150.27
Preprocessed AB.[direct]	137.41
Preprocessed AB.[age]	135.98
Preprocessed AB.[refer]	130.23
Preprocessed AB.[language_development]	128.61
Preprocessed AB.[hear_aid]	128.15
Preprocessed AB.[detection]	123.85
Preprocessed AB.[place]	119.44
Preprocessed AB.[base]	117.42
Preprocessed AB.[point]	116.75
Preprocessed AB.[listen]	115.41
Preprocessed AB.[excellent]	110.98
Preprocessed AB.[widely]	110.75
Preprocessed AB.[English]	110.69
Preprocessed AB.[psychological]	109.72

**Table 6:** Some of the abstract *n*-grams with negative weights.

Feature	Weight
Preprocessed AB.[amplitude]	-77.38
Preprocessed AB.[regard]	-77.63
Preprocessed AB.[world]	-77.78
Preprocessed AB.[occur]	-78.17
Preprocessed AB.[normal]	-81.00
Preprocessed AB.[aid_condition]	-82.22
Preprocessed AB.[profound_deafness]	-82.57
Preprocessed AB.[child_use]	-82.95
Preprocessed AB.[potential_record]	-85.43
Preprocessed AB.[overall]	-87.01
Preprocessed AB.[child_implant]	-90.88
Preprocessed AB.[outcome]	-93.81
Preprocessed AB.[month_implantation]	-95.26
Preprocessed AB.[receptive]	-95.41
Preprocessed AB.[frequency_information]	-96.82
Preprocessed AB.[treat]	-96.91
Preprocessed AB.[distort]	-102.61
Preprocessed AB.[achieve]	-107.08
Preprocessed AB.[implant_year]	-111.90
Preprocessed AB.[post]	-117.16
Preprocessed AB.[old]	-117.89
Preprocessed AB.[site]	-124.55

**Table 7:** Using different models to predict the total citations using the paper abstract.

Algorithm	Mean absolute error	Root mean squared error	Relative absolute error	Relative squared error	Coefficient of determination
Linear regression	51.49	68.56	1.25	1.30	-0.30
Boosted decision tree regression	47.87	66.00	1.16	1.21	-0.21
Decision forest regression	42.75	63.53	1.04	1.12	-0.12
Neural network	40.48	62.76	0.98	1.09	-0.09

**Table 8:** Error in citation count.

Error	Percentage of citation range (523 citations)	Paper count	Percentage of testing papers (145 papers)
≤10 citations	1.9%	46 papers	31.72%
≤40 citations	7.6%	93 papers	64.13%
≤80 citations	15.29%	127 papers	87.58%
≤100 citations	19.12%	135 papers	93.1%

**Table 9:** Using different models to predict the total citations using the paper authors.

Algorithm	Mean absolute error	Root mean squared error	Relative absolute error	Relative squared error	Coefficient of determination
Linear regression	50.12	69.58	1.049	1.12	-0.12
Boosted decision tree regression	45.34	65.79	0.949	1.00	-0.00
Decision forest regression	46.94	67.36	0.98	1.05	-0.05
Neural network	49.84	70.19	1.04	1.14	-0.14

**Table 10:** Error in citation count.

Error	Percentage of citation range (523 citations)	Paper count	Percentage of testing papers (150 papers)
≤10 citations	1.9%	23 papers	15.33%
≤40 citations	7.6%	90 papers	60%
≤80 citations	15.29%	130 papers	86.66%
≤100 citations	19.12%	136 papers	90.66%

**Table 11:** The best algorithms and the corresponding RMSE.

Feature	Best algorithm	Root mean squared error
Title	Decision forest regression	69.45
Abstract	Neural network	62.76
Authors	Boosted decision tree regression	65.79

**Table 12:** Number of *n*-grams for each feature.

The feature used in prediction	*n*-grams
Title	164
Abstract	1714
Authors	94

## Data Availability

The data used to support the findings of this study are available from the corresponding author upon request.
